The article "Study on the Potential Molecular Mechanism of Xihuang Pill in the Treatment of Pancreatic Cancer Based on Network Pharmacology and Bioinformatics" was published in 2022. Journal: Evid Based Complement Alternat Med.

# Study on the Potential Molecular Mechanism of Xihuang Pill in the Treatment of Pancreatic Cancer Based on Network Pharmacology and Bioinformatics

**DOI:** 10.1155/2022/4651432

**Published:** 2022-04-11

**Authors:** Jing Wang, Yaxing Zhang, Qiuyuan Wang, Luyao Wang, Peitong Zhang

**Affiliations:** ^1^Guang Anmen Hospital, China Academy of Traditional Chinese Medicine, Beijing 100053, China; ^2^Graduate School, Beijing University of Chinese Medicine, Beijing 100029, China; ^3^Zhejiang Chinese Medical University, Hangzhou, Zhejiang 310053, China; ^4^Department of Orthopaedics, China-Japan Friendship Hospital, Beijing 100029, China

## Abstract

**Objective:**

We aimed to analyze the possible molecular mechanism of Xihuang pill (XHP) in the treatment of pancreatic cancer based on methods of network pharmacology, molecular docking, and bioinformatics.

**Methods:**

The main active components and targets were obtained through the TCMSP database, the BATMAN-TCM database, and the Chemistry database. The active ingredients were screened according to the “Absorption, Distribution, Metabolism, Excretion” (ADME) principle and supplemented with literature. We searched GeneCards, OMIM, TTD, and DrugBank databases for pancreatic cancer targets. The targets of disease and ingredients were intersected to obtain candidate key targets. Then, we constructed a protein-protein interaction (PPI) network for protein interaction analysis and a composition-key target map to obtain essential effective ingredients. Metascape was used to perform functional enrichment analysis to screen critical targets and pathways. The expression and prognosis of key targets were examined and analyzed, and molecular docking was carried out.

**Results:**

A total of 52 active ingredients of XHP, 121 candidate targets, and 52 intersecting targets were obtained. The core active ingredients of XHP for the treatment of pancreatic cancer were quercetin, 17-*β*-estradiol, ursolic acid, and daidzein. The core targets were EGFR, ESR1, MAPK1, MAPK8, MAPK14, TP53, and JUN, which were highly expressed genes of pancreatic cancer. Among them, EGFR and MAPK1 were significantly correlated with the survival of pancreatic cancer patients. The key pathway was the EGFR/MAPK pathway. The molecular docking results indicated that four active compositions had good binding ability to key targets.

**Conclusion:**

The molecular mechanism of XHP for the treatment of pancreatic cancer involved multiple components, multiple targets, and multiple pathways. This research theoretically elucidated the ameliorative effect of XHP against pancreatic cancer and might provide new ideas for further research on the treatment of pancreatic cancer.

## 1. Introduction

Pancreatic cancer is one of the most lethal malignant neoplasms, which causes over 331000 deaths per year worldwide and ranks as the seventh most common cancer death [1]. Surgical resection with the addition of chemotherapy and radiotherapy plays an important role in the management of pancreatic cancer. Despite advances in chemotherapy, the overall 5-year survival rates ranged from 2% to 9% and remained relatively unchanged over the past several decades [2]. Therefore, new treatment strategies are needed for pancreatic cancer to achieve longer survival. Traditional Chinese medicine (TCM) has been applied clinically in China for more than a thousand years. As one of the most popular complementary and alternative medicine modalities in China, TCM has been gradually accepted due to its prominent efficacy and less toxicity.

Xihuang pill (XHP), as a famous TCM formula, has been used to clear heat, relieve toxicity, and expel stasis of blood since the Qing dynasty. It is composed of Niu Huang (*Bovis Calculus*), She Xiang (*Moschus*), Ru Xiang (*Olibanum*), and *Mo Yao* (*Commiphora myrrha*). Modern pharmacological studies demonstrated that XHP could enhance chemosensitivity, relieve side effects of conventional therapies, and ameliorate prognosis when used as a complementary therapy [3–6]. XHP exerts antitumor effects in multiple ways including inhibiting the growth, invasion, and metastasis of tumor cells, preventing angiogenesis, and improving the tumor immune microenvironment [7]. However, the chemical and pharmacological foundations of XHP in inhibiting pancreatic cancer have not been evaluated with appropriate approaches yet.

Because of the complexity in the compositions of TCM, conventional pharmacological approaches may not be applicable to TCM research. Network pharmacology, based on system biology, emphasizes the multipath regulation of signal pathways by drugs and studies the gene regulation and protein interaction networks of complex diseases [8–10]. This “multigene-multitarget-complex disease” research model is consistent with the holistic concept of TCM treatment.

Bioinformatics is a discipline that uses applied mathematics, informatics, computer science, and other methods to study biological problems [11, 12]. Biological data such as DNA sequence, gene expression, and protein structure will be integrated, screened, processed, and calculated in order to extract useful biological information from large data, and analyze the biological information of expressed structure and function from the level of nucleic acid and protein, which is helpful to explore the biological pathways and networks.

Thus, based on the theoretical basis of network pharmacology and bioinformatics, this study explored the potential mechanism of XHP in the treatment of pancreatic cancer.

## 2. Materials and Methods

### 2.1. Acquisition of Active Ingredients and Targets

The Traditional Chinese Medicine Systems Pharmacology Platform [13] (TCMSP) (https://tcmspw.com/tcmsp.php) was used to search the active ingredients of XHP. The filter criteria were oral bioavailability (OB) ≥ 30% and drug-likeness (DL) ≥ 0.18 according to the “Absorption, Distribution, Metabolism, and Excretion” (ADME) principle. Only when the ingredients in XHP met both of these two prerequisites were they considered as possible active ingredients of XHP. For the herbs in XHP whose information of active ingredients cannot be acquired from TCMSP database, they were screened in other authoritative websites such as BATMAN-TCM database [14] (http://bionet.ncpsb.org/batman-tcm/) and Chemistry database (http://www.organchem.csdb.cn). A literature search was also conducted to get supplements for the active ingredients of XHP which have been reported to have definite pharmacologic action for pancreatic cancer. The target information of the active ingredients was mainly acquired from the TCMSP database and was recorded by the DrugBank database [15, 16]. Then we accomplished the standardization of gene names and corresponding information search through the UniProt database [17] (https://www.uniprot.org/).

### 2.2. Gain the Targets of Pancreatic Cancer

We searched the keyword “pancreatic cancer” in GeneCards [18] (https://http://www.genecards.org/), Online Mendelian Inheritance in Man [19] (https://www.omim.org/), Therapeutic Target Database [20] (http://db.idrblab.net/ttd/), and DrugBank database (https://go.drugbank.com/) to comprehensively find relevant targets of pancreatic cancer. After getting the target information of pancreatic cancer, duplicate removement was conducted. Among them, the screening of the targets from the GeneCards database was conducted according to the median of their relevance to pancreatic cancer.

### 2.3. Target Intersection Analysis

The *R* package “VennDiagram” was applied to map and intersect the targets of pancreatic cancer and targets of active ingredients in RStudio software, and the result was shown through a Venn diagram for a clear display.

### 2.4. PPI Network Construction

We employed the STRING [21] (https://string-db.org/) website to construct the PPI network analysis by choosing “multiple sequences” in function units and setting “Homo sapiens” as the organism specie with the interaction confidence retaining the acquiescent value of 0.4. The result of the PPI network analysis was saved as a TSV document and was imported into Cytoscape 3.8.1 software. Then, the MCODE plug-in [22] was used for topology analysis to extract the key gene module. After obtaining the key genes, we found out the corresponding active ingredients of XHP and constructed the “composition-target” network diagram.

### 2.5. Enrichment Analysis

Metascape [23] (https://metascape.org/) was used for the gene enrichment analysis to get the function of the targets in the key gene module and to explore the biological process and corresponding pathways. Results were expressed as logP values, reflecting the significance of protein biological functions, and all results were considered significant at *P* < 0.01.

### 2.6. Expression and Survival Analysis of the Key Targets

GEPIA (Gene Expression Profiling Interactive Analysis) (http://gepia.cancer-pku.cn/) [24] is a database to take an overview of the profiles of the studied genes in different tumors. Here we used the database to investigate the different expression levels of every single key target in pancreatic cancer and normal tissue. The cutoff value of |Log2FC| was set to be 1, and the *p* value cutoff value was set to be 0.01. The KM plotter (https://kmplot.com/analysis/) [25] was employed to assess the prognostic value of different key targets, according to the gene expression in tumor samples of 177 patients with pancreatic cancer, the samples were divided into high expression group and low expression group for survival analysis. The Kaplan–Meier method was used to compare the survival data of the two groups. All the results were statistically significant when *p* < 0.05.

### 2.7. Molecular Docking

Molecular docking is a reliable approach for drug design based on the characteristics of receptors and the interaction between receptors and ligands, and ligands are typically drug molecules. We searched the 3D structures of the proteins corresponding to the key targets and used them as receptors for further docking. The ligands were the main active ingredients of XHP which we obtained after screening by the above methods, which were potentially effective for the treatment of pancreatic cancer. After that, CB-Dock (http://cao.labshare.cn/cb-dock/) [26] was used for molecular docking.

## 3. Results

Bezoar and musk have different main components due to different varieties, but it is not documented in detail in the TCMSP database, and musk is not recorded in the database. Therefore, we referred to relevant literature and databases to confirm the components of cultured bezoar in vitro and artificial musk in XHP sold commercially. Moreover, in the published literature, no pharmacological effect directly related to pancreatic cancer was collected in bezoar, musk, frankincense, and myrrh. In addition, the ingredients of XHP that did not meet the filter criteria in the TCMSP database were also included in this study because the related targets information of which in the database was linked to pancreatic cancer.

After normalization of the target names in the UniProt database and duplication omitting, there were 6 active ingredients and 24 related targets in bezoar, 6 active ingredients, and 55 related targets in musk. In frankincense, six active ingredients were identified, corresponding to 35 targets. We found 35 active ingredients and 93 corresponding targets in myrrh, respectively. After removing duplicates, we collected 52 active ingredients in the XHP and a total of 121 related target genes. Among them, bezoar contained CLRs (Mol ID : MOL000953) as same as musk. The results are presented in Table 1.

Through four consecutive screenings, 731 pancreatic cancer targets were identified in the GeneCards database. Other targets information obtained from the OMIM and TTD disease databases were combined, resulting in 1224 disease targets after removing duplicates. After Venn diagram analysis, 52 intersection targets between XHP and pancreatic cancer were finally confirmed (Figure 1). The results of interaction mapping of intersection target proteins constructed by the STRING database are shown in Figure 2. Nodes represent all proteins produced by a single gene locus, and lines represent proteins that collectively contribute to function, while the color of lines represents sources of evidence for drawing associations, such as purple for experimental validation, yellow for text mining, and black for coexpression among proteins.

We downloaded the interaction network in TSV files and imported it into Cytoscape software. An interactive network consisting of 52 points and 533 edges was obtained. The Mcode plug-in was utilized to acquire the key module. The Mcode is an algorithm that calculates the information of individual nodes in the network. The final module, obtained after processing according to the parameters of the nodes, is the key functional module in the interaction network. The results yielded a total of 27 key targets, which were ranked according to the degree value, as shown in Table 2.

An ingredient-key target network diagram was constructed in Cytoscape software, as shown in Figure 3. Nodes are for each target and ingredient, and lines represent correlations between nodes. The greater the degree value of a node, the darker the color, which indicates the degree of connectivity is greater. Therefore, the key active ingredients were quercetin, 17-*β*-estradiol, ursolic acid, and daidzein.

The Metascape platform is a gene functional annotation analysis tool that enables cognition of gene and protein function by applying bioinformatic analysis methods to analyze bulk genes and proteins. After importing the 27 potential key targets of XHP for pancreatic cancer into the Metascape platform, Kyoto Encyclopedia of Genes and Genomes (KEGG) pathway enrichment analysis and gene ontology (GO) analysis were performed, respectively. The results of GO analysis included three sections: cellular components (CC), molecular functions (MF), and biological processes (BP). The cellular component result section reflects the location in the cell of the gene, the molecular function result section reflects the effect of a single gene product, and the biological process result section comprises various biological processes in which genes are involved, such as apoptosis and so on.

Further identification of the module yielded key functional modules (Figure 4). The module included EGFR, MAPK1, MAPK8, MAPK14, TP53, ESR1, and JUN genes. The enrichment analysis results were ranked according to logP value, and the top 20 results were selected and presented as a bubble plot (Figure 5). The color of the bubbles from red to green represented the LogP value from small to large, and the larger the bubble is, the more genes are enriched in this pathway.

Finally, the cellular components of the genes involved in the vesicle lumen, membrane rafts, extracellular matrix, adherent junctions, the outer side of the plasma membrane, and so on. The molecular functions included cytokine receptor binding, heme binding, MAP kinase activity, serine-type endopeptidase activity, phosphatase binding, and so on. Biological processes involved positive regulation of cell migration, positive regulation of the MAPK cascade, positive regulation of protein serine/threonine kinase activity, response to hypoxia, and apoptosis. The biological pathways mainly included pathways in cancer, the MAPK signaling pathway, the NF-*κ*B signaling pathway, the JAK-STAT signaling pathway, and the IL-17 signaling pathway. Taking the MAPK signaling pathway as an example, the mechanism and potential targets of this pathway are shown in Figure 6. Yellow nodes represent the enzymes or other compounds related to potential targets.

As shown in Figure 7 and Figure 8, compared with the expression of key targets in normal tissues, EGFR, ESR1, MAPK1, MAPK8, MAPK14, TP53, and JUN genes in pancreatic cancer were highly expressed. The expression differences of MAPK1, MAPK8, MAPK14, and TP53 were obvious, followed by EGFR and JUN, and the target with the least expression difference was ESR1. The Kaplan–Meier analysis showed that the expressions of EGFR, MAPK1, MAPK14, and TP53 were negatively correlated with survival time, while the expressions of ESR1, MAPK8, and JUN were positively correlated with survival time. Besides, there was no statistical significance in the results of ESR1, MAPK8, MAPK14, TP53, and JUN (*P* > 0.05).

In molecular docking, EGFR and MAPK1 were used as receptors, and the active ingredients, quercetin, 17-*β*-estradiol, ursolic acid, and daidzein, were used as ligands for docking to verify the potential active components and targets of XHP on pancreatic cancer (Table 3 and Figure 9). The results indicated good binding ability, confirming the effectiveness and authenticity of the therapeutic components and targets.

## 4. Discussion

XHP has therapeutic effects on diverse tumors. It is widely used as a supplementary drug in the treatment of a variety of malignant tumors in China, such as pancreatic cancer [6], lung cancer [27], gastric cancer [28], and breast cancer [29]. However, the underlying mechanisms of XHP treating cancers remain unclear. Pancreatic cancer is a solid tumor with a very poor prognosis, and the treatment of which is still extremely difficult. Therefore, it is significant to find out the pharmacological mechanisms of XHP for the treatment of pancreatic cancer.

TCM is rooted in tens of centuries of clinical practices. Its curative effects are closely associated with the interaction of multiple ingredients, targets, and pathways. One of the difficulties in the pharmacological study of TCM is the numerous active components. Thus, network pharmacology has the advantage of searching for the key effective ingredients of traditional Chinese herbs, elucidating the regulation principles of complex molecules by constructing and establishing the systematic network of compound-protein and gene-disease [30].

In our present study, we applied the pharmacological method to predict and elucidate the potential molecular mechanisms of the action of XHP on pancreatic cancer. In the XHP active components and corresponding targets results, a total of 52 bioactive compounds and 121 targets in the XHP were obtained. There were 4 compounds including quercetin, ursolic acid, daidzein, and 17-beta-estradiol identified as the potential active ingredients of XHP, of which the biological activities against pancreatic cancer were reported previously [31]. For example, quercetin can inhibit the expression of the receptor for advanced glycation end products (RAGE), inhibit the PI3K/AKT/mTOR axis, regulate the death of pancreatic cancer cells, and increase the chemosensitivity of gemcitabine [32]. Ursolic acid also has an effect on increasing gemcitabine (GEM) chemosensitivity in pancreatic cancer cells possibly by triggering endoplasmic reticulum (ER) stress, activating apoptosis- and autophagy-related pathways, and decreasing the expression of RAGE [33]. In addition, an ex vivo assay shows that daidzein exhibits cytotoxic effects and genotoxic effects on human pancreatic cancer cell lines in a dose-dependent manner [34]. Besides, it is reported that the addition of *β*-estradiol with chemotherapeutic drugs increases chemosensitivity to pancreatic ductal adenocarcinoma [35]. Therefore, the abovementioned research studies indicate that many bioactive ingredients of XHP possess diverse effectiveness for treating pancreatic cancer.

The results of KEGG and GO enrichment analysis show that the therapeutic effect of the XHP in pancreatic cancer is mainly involved in the MAPK pathway, the NF-*κ*B pathway, IL17 signaling, pathways in cancer, etc. These results are in agreement with other results suggesting that Integrin/EGFR-ERK/MAPK signaling promotes the growth and metastasis of pancreatic tumors [36]. Besides, the NF-*κ*B pathway, as an important inflammatory mediator, is constitutively activated in pancreatic cancer and plays a crucial role in the development, progression, and drug resistance of pancreatic cancer [37]. IL17/IL17RA signaling is involved in pancreatic tumorigenesis, and IL17 blockade ameliorates PD-1 sensitivity [38].

Subsequently, the function gene module was identified through Metascape, which is a potential target module of XHP for pancreatic cancer. The gene module includes EGFR, ESR1, MAPK1, MAPK8, MAPK14, TP53, and JUN. The analysis results of the expression level verified that the key genes listed above were upregulated in pancreatic cancer samples compared with control samples. Further survival analysis of the Kaplan–Meier estimate showed that EGFR and MAPK1 were negatively correlated with survival time, which was statistically significant.

Furthermore, the molecular docking assay in this study showed that the four key active ingredients of XHP had good binding ability to key targets (EGFR and MAPK1). The CB-Dock website can predict the binding site of a given protein, calculate the center and size using a new curvature-based cavity detection method, and perform AutoDock Vina molecular docking. The lower the Vina score value, the higher the affinity between the receptor and the ligand. The docking results indicated that 17-beta-estradiol was verified the strongest binding activity with both EGFR and MAPK1 among the four potential key active ingredients.

Combining the enrichment and module analysis, the inhibition of the EGFR/MAPK pathway by XHP should be noted. EGFR is a transmembrane protein closely related to multiple pathological processes such as the proliferation, invasion, and metastasis of pancreatic cancer cells. Clinical studies have shown that the overexpression of EGFR could shorten the average overall survival rate of patients after PDAC resection and can be used as an independent predictor [39]. Accumulating evidence demonstrated that MAPK signaling promotes pathogenesis and biochemical progress of tumor cells [40]. MAPK cascades are substrates of activated EGFR. XHP could possibly inhibit EGFR and the downstream MAPK pathway.

High-throughput omics techniques, including proteomic and transcriptomic analysis, have enabled further comprehension of the TCM [41]. Though we predicted the possible targets by XHP by network pharmacology and molecular docking, the results are predictions after all. And for the next step, we intend to use XHP to treat pancreatic cancer both in vivo and in vitro experimental models, analyzing expression levels of protein and mRNA level by transcriptomics and proteomics studies.

## 5. Conclusion

In conclusion, this comprehensive network pharmacological analysis proposes numerous testable surmises about the potential molecular mechanisms of XHP formula for the treatment of pancreatic cancer and predicts that quercetin, 17-*β*-estradiol, ursolic acid, and daidzein are potential bioactive ingredients of XHP, which act on key genes such as EGFR and MAPK1 and regulate many pathways (EGFR/MAPK pathway, IL-17 signaling pathway, NF-*κ*B pathway, pathways in cancer, etc.). It also should be noted that the XHP formula possibly exhibits an anti-tumor effect by regulating multiple biological pathways. The prediction results theoretically elucidated the ameliorative effect of XHP against pancreatic cancer and might facilitate further research on the mechanism of XHP or its bioactive compounds as an alternative therapy for pancreatic cancer.

## Figures and Tables

**Figure 1:** Venn diagram of intersection targets (PC: pancreatic cancer).

**Figure 2:** Protein interaction diagram.

**Figure 3:** Composition-key target network diagram.

**Figure 4:** Key functional modules.

**Figure 5:** Functional enrichment bubble diagrams: (a) Go - CC diagram; (b) GO - MF diagram; (c) GO - BP diagram; (d) KEGG diagram.

**Figure 6:** MAPK signal pathway diagram.

**Figure 7:** Expression level of key targets.

**Figure 8:** Survival analysis of key targets.

**Figure 9:** Docking modes: (a) EGFR-quercetin; (b) EGFR-17-beta-estradiol; (c) EGFR-ursolic acid; (d) EGFR-daidzein; (e) MAPK1- quercetin; (f) MAPK1-17-beta-estradiol; (g) MAPK1-ursolic acid; (h) MAPK1- daidzein.

**Table 1:** List of active ingredients in XHP.

Herb	Mol ID	Molecule name	Targets
SHE XIANG	MOL001232	Testosterone	3
	MOL010919	17-Beta-estradiol	38
	MOL000737	Morin	6
	MOL002361	Estragole	14
	MOL004783	N-Nonane	2
	MOL000953	Cholesterol	3
NIU HUANG	MOL008838	methyl(4R)-4-[(3R,5S,7S,8 R,9S,10S,12S,13 R,14S,17 R)-3,7,12-trihydroxy-10,13-dimethyl-2,3,4,5,6,7,8,9,11,12,14,15,16,17-tetradecahydro-1h-cyclopenta[a]phenanthren-17-yl]pentanoate	2
	MOL008839	Methyl desoxycholate	3
	MOL008845	Deoxycholic acid	4
	MOL008846	ZINC01280365	5
	MOL000953	CLR	3
	MOL000511	Ursolic acid	19
RU XIANG	MOL001215	Tirucallol	2
	MOL001241	O-acetyl-*α*-boswellic acid	1
	MOL001243	3alpha-hydroxy-olean-12-en-24-oic-acid	6
	MOL001255	Boswellic acid	2
	MOL001295	Phyllocladene	1
	MOL000390	Daidzein	27
MO YAO	MOL001001	Quercetin-3-O-*β*-D-glucuronide	3
	MOL001002	Ellagic acid	10
	MOL001004	Pelargonidin	11
	MOL001006	Poriferasta-7,22e-dien-3beta-ol	3
	MOL001009	Guggulsterol-VI	1
	MOL001013	Mansumbinoic acid	1
	MOL001026	Myrrhanol C	4
	MOL001028	(8R)-3-oxo-8-hydroxy-polypoda -13E,17 E,21-triene	2
	MOL001029	Myrrhanones B	2
	MOL001031	Epimansumbinol	4
	MOL001033	Diayangambin	5
	MOL001040	(2R)-5,7-dihydroxy-2-(4-hydroxyphenyl) chroman-4-one	6
	MOL001045	(13E,17 E,21E)-8-hydroxypolypodo-13,17,21-trien-3-one	2
	MOL001046	(13E,17 E,21E)-polypodo-13,17,21-triene-3,18-diol	1
	MOL001049	16-Hydroperoxymansumbin-13(17)-en-3*β*-ol	2
	MOL001052	Mansumbin-13(17)-en- 3,16-dione	6
	MOL001061	(16S, 20R)-dihydroxydammar-24-en-3-one	5
	MOL001062	15*α*-hydroxymansumbinone	5
	MOL001063	28-Acetoxy-15*α*-hydroxymansumbinone	4
	MOL001095	Isofouquierone	2
	MOL001126	[(5aS,8aR,9R)-8-oxo-9-(3,4,5-trimethoxyphenyl)-5,5a,6,9-tetrahydroisobenzofurano[6,5-f] [1,3] benzodioxol-8a-yl] acetate	16
	MOL001131	Phellamurin_qt	6
	MOL001138	(3R,20S)-3,20-dihydroxydammar- 24-ene	6
	MOL001156	3-Methoxyfuranoguaia-9- en-8-one	9
	MOL001175	Guggulsterone	5
	MOL000358	Beta-sitosterol	21
	MOL000449	Stigmasterol	23
	MOL000490	Petunidin	7
	MOL000098	Quercetin	55
	MOL000988	4,17(20)-(cis)-pregnadiene-3,16-dione	2
	MOL000996	Guggulsterol IV	3
	MOL001125	Erlangerin B	2
	MOL001127	Erlangerin D	7
	MOL000254	Eugenol	25
	MOL000978	Furanoeudesma- 1,4-diene-6-one	11

**Table 2:** Key targets.

Name	Closeness centrality	Degree	Betweenness centrality
TP53	0.85	42	0.068810131
VEGFA	0.836065574	41	0.056756149
IL6	0.796875	38	0.05317606
MAPK1	0.796875	38	0.043544924
EGF	0.784615385	37	0.037239889
EGFR	0.784615385	37	0.043334685
JUN	0.76119403	35	0.022646029
MAPK8	0.76119403	35	0.024236994
TNF	0.739130435	33	0.01515152
ESR1	0.739130435	33	0.043118785
PTGS2	0.739130435	33	0.013562229
IL1B	0.728571429	32	0.012370454
MMP2	0.718309859	31	0.010559301
MAPK14	0.708333333	30	0.012303754
CAT	0.698630137	30	0.05575807
CCL2	0.708333333	30	0.007732274
MMP1	0.662337662	26	0.017930964
MMP3	0.662337662	26	0.016948756
MPO	0.671052632	26	0.016875167
IFNG	0.671052632	26	0.006005576
NGF	0.662337662	25	0.006541835
IL2	0.662337662	25	0.00545143
CXCL12	0.653846154	25	0.004267719
CXCR4	0.6375	23	0.003965538
HMOX1	0.64556962	23	0.00604897
PLAU	0.62195122	21	0.001768495
NOS2	0.593023256	17	7.63E-04

**Table 3:** Docking results of key active ingredients and key targets.

	Quercetin	17-Beta-estradiol	Ursolic acid	Daidzein
	Vina score	Vina score	Vina score	Vina score
EGFR	-8	-8.8	-8.3	-7.8
MAPK1	-8.5	-8.9	-8.8	-7.9

## Data Availability

All the data and materials used in the current study are available from the corresponding author upon reasonable request.
